The article "Analysis of the Effect of the Stability of Athletes' Psychological Quality on Sports Basketball Games" was retracted in 2023. Reasons: signs of a paper mill; suspected computer-generated content; unreliable results or conclusions; lack of ethics approval or compliance.

# Analysis of the Effect of the Stability of Athletes' Psychological Quality on Sports Basketball Games

**DOI:** 10.1155/2022/8624803

**Published:** 2022-08-24

**Authors:** Xin Zhang, Xiaoyun Zeng

**Affiliations:** ^1^Sport Department, Xi'an Kedagaoxin University, Xi'an, Shaanxi 710109, China; ^2^School of Physical Education, Xi'an University of Architecture and Technology, Xi'an, Shaanxi 710055, China

## Abstract

Enthusiasm for sports competitions is consistently high. In sports competitions, athletes not only need to have superb skills but also need a strong psychological quality. Usually, athletes with high psychological quality can make their technical level outstanding; on the contrary, for athletes with low psychological quality, even if the level of competition is very high, it is difficult to achieve excellent results. This study analyzes the data of basketball players to study the influence of the stability of different players' psychological quality on the performance of basketball games. The “mental state” of basketball players is negatively correlated with their performance in basketball games, and the players' psychology often shows signs of tension during basketball games. This tension is the result of a variety of psychological effects, and the number of times of tension is different under different psychological quality stabilities. The experimental analysis results of this study show that through the data analysis of the psychological factors affecting basketball players, the key factors affecting their psychology have been explored, and strategies and methods that can effectively cultivate the psychological quality of basketball players have been found, in order to provide a reference for improving the psychological quality of basketball players.

## 1. Introduction

With the continuous development of science and technology, the intensity and visual enjoyability of sports are also increasing. How to improve the performance of sports athletes becomes an important issue [1, 2]. People can build up a good physique through sports, and can also increase physical knowledge and enrich physical activities by watching sports games [3]. The high-frequency holding of the Asian Games, Olympic Games, and other competitions has made competitive sports develop rapidly, typically team-based competitive competitions such as football, basketball, and volleyball [4, 5]. As an important ball game, basketball is actually a diversified transformation from the traditional “futsal” and “three-player system” to beach basketball. In the current basketball game, the grasp of “air supremacy” often takes the main advantage in confrontation, especially when the level of competition is almost the same, and the advantage of “air supremacy” is more prominent. As a sport with strong competitive skills, basketball is gradually developing in the direction of “fast, diverse, high and complete,” and as a participating athlete, the most important thing is the physical quality of basketball players, while mastering higher competitive skills [6, 7]. Whether physical fitness is good or not is the relevant basis for mastering new skills, techniques, and tactics, and is the basis for ensuring certain results in the corresponding competition [8, 9]. In order to occupy a certain net advantage in competitive competitions and take the initiative in the competition, many coaches choose athletes with higher heights when selecting backup athletes, so that they can occupy the main height advantage in the process of net competitions. On the basis of height selection, many coaches conduct targeted psychological quality training by learning the skills of excellent basketball players, and at the same time, they analyze the weaknesses and deficiencies of the players based on the continuous watching of the game and review of the game, so as to enhance their skills in a targeted manner [10, 11]. Therefore, basketball needs scientific psychological training modes and methods to improve and exercise the skills and techniques of athletes, which are extremely important.

In view of these needs and deficiencies, based on the psychological quality stability model, we try to sort out the business logic of basketball. By analyzing the evaluation and analysis of the movement of athletes' psychological quality training in competition, the corresponding multivariate analysis of physical quality is constructed, to explore and analyze the development model of basketball players' physical bounce, aiming to provide a basis and analysis for basketball players' bounce analysis and scientific implementation of psychological quality training. In the 1980s, foreign research on the psychological stress of basketball players on the court has begun, but Chinese research on this aspect has mainly started in recent years, and it is still in the exploratory stage. It is mainly descriptive and explanatory research on the tension phenomenon of players, but there are few experimental researches. The training of psychological quality is a special endurance quality that combines the two elements of endurance and speed and combines the comprehensive influencing factors of endurance and speed. The training of mental quality is the dual embodiment of muscle speed and endurance. For an athlete, the greater the endurance used when the action is completed, the faster the corresponding speed, and the greater the speed and endurance displayed. Explosive force is an important manifestation of psychological quality. According to the specific load influencing factors of rapid psychological quality training, explosive force and psychological quality training are carried out, and the load is adjusted, so as to carry out a comprehensive analysis of maximum endurance, explosive force training, and psychological quality training [12–14]. The methods of training psychological quality mainly include: one is to promote individual muscle group training or auxiliary movements of special movements through general training exercises, so relatively speaking, the load is larger; the other is that through special training exercises, the space-time structure of the exercise and the working method of the muscles can be closer to the real competition, especially through the playback of the competition schedule, the replay can be achieved with a small load. In the process of training basketball players' psychological quality, it is necessary to combine the degree of cooperation and enthusiasm of the athletes to evaluate the effect of psychological training. If basketball players are skeptical about psychological training, it will lead to difficulty in controlling their psychological training. Therefore, basketball players also need to correct their training thinking, so as to ensure that their psychological training can be improved to the greatest extent.

With the continuous development of the social economy, sports have become one of the important daily necessities. Therefore, it is extremely important to focus on sports psychological quality training and improve basketball performance. In view of these needs and certain limitations, based on the psychological quality stability model, this study analyzes the effectiveness of the psychological quality training of basketball players by sorting out the psychological quality training methods of basketball players, and deeply analyzes the training. Relationship between the psychological influencing factors of physical fitness and other psychological quality training, and corresponding tests are carried out to realize the analysis and dissection of the competition, and realize the statistical analysis of the calculation of the model results, aiming to analyze the effective psychological quality training programs of athletes. The simulation results show that the psychological quality stability model proposed in this study is effective, has high stability and prediction accuracy, and can provide a theoretical reference for the development of basketball players' psychological quality, so as to further improve the performance of sports psychological quality training.

## 2. Objects and Methods of Research

### 2.1. Research Object

The experimental target selected in this study is basketball players in a city's colleges and universities, and a total of 126 questionnaires are distributed. Among them, there are 108 valid questionnaires, involving 67 boys and 41 girls, the age is mainly 18–23 years old, and the sports years are 4–10 years.

### 2.2. Research Method

#### 2.2.1. Evaluation of Basketball Performance

The current evaluation of basketball players' performance is mainly divided into two methods: subjective and objective. According to the objective evaluation method, set shot or non-set shot is usually used. Since basketball has a high technical content, it can effectively reflect the competitive ability of basketball players. Therefore, Therefore, research scholars of China and other countries generally use the method of testing the number of successful shots of athletes to evaluate their game performance, which can roughly evaluate the skill level of basketball players. The subjective evaluation method is mainly combined with the self-satisfaction evaluation of basketball players. In the experiment process of this paper, according to the different stabilities of athletes' psychological quality, appropriate methods of subjective evaluation of athletes are selected. Using the Likert equidistant evaluation method to calculate the score, 1–5 is adopted to score the satisfaction performance of basketball players. The higher the score, the higher the degree of satisfaction. Among them, the score, 1 number “1” means very dissatisfied, and “5” means very satisfied.

#### 2.2.2. Contents of the Psychological Quality Assessment Questionnaire for Athletes

The content of the questionnaire on the stability of mental quality of sports athletes is mainly divided into basic scenarios and combined scenarios [15, 16]. The basic scenario mainly sets 15 related questions. The Likert equidistant evaluation method is used to calculate the score, and 1–5 is used to score the satisfaction performance of basketball players. The higher the score obtained, the better the performance of the basketball player; the combined scenarios are set as a combination of 15 different scenarios. In order to ensure the validity of the questionnaire survey, the questionnaire survey set up in this paper uses the evaluation method of reliability and validity. For the 15 basic questions involved in the questionnaire, the KMO test method is used, the value of the calculated result is 0.787, which is relatively high, indicating that there are influential factors in the 15 questions set, and then Bartlett's spherical test is used, the significant value obtained by this test is high, which can indicate that the method of factor analysis can be used for the questionnaire survey in this paper. Through using SPSS software, a total of six eigenvalues exceeding 1 can be obtained, and the total contribution rate can reach 96.15%, indicating that six influencing factors can be selected, which are defined as game time, game process, criticality, psychological status, and opponent skill level and paper game of home and away.

In order to test the reliability of the questionnaire, the SPSS software is used to test the split-half reliability of the questionnaire, and the test results can reach 0.768–0.832, which indicates that the reliability of the questionnaire is very high. The validity of the questionnaire is usually the construct validity, and the correlation between the factors can be analyzed by using the factor analysis method. Through the analysis results, it can be seen that the correlation between the factors is low, the test value is maintained between 0.228 and 0.303, and the correlation between the factors and the total summary is very large, indicating that the factors do not belong to different sets, and that the construct validity of the questionnaire is good.

## 3. Results and Analysis

### 3.1. The Influence of Psychological Quality Stability on Competition Performance

Many factors affect the stability of psychological quality in basketball games, such as the progress of the basketball game and the difference in score. These factors can cause mood fluctuations in basketball players, which in turn can lead to changes in basketball game results. The goal of the experiment in this paper is to test the degree of influence that leads to the stability of athlete's psychological quality on the results of the game, by selecting 15 influencing factors and six influencing factors of psychological quality stability, as shown in Table 1.

According to the test results in Table 1, it can be seen that the value of the influencing factor of the psychological quality stability of basketball players is 6, indicating that the psychological quality stability of athletes greater than 6 is poor. For example, according to the analysis of basketball game time, it can be mainly divided into three stages: the initial stage of the game, the process of the game and the end of the game; from the score of the game, it can be seen that there is a stage of outscore, a stage with a lower score, and a stage with a similar score. According to the test results in Table 2, the scores of the competition under the stability of different athletes' psychological quality, the numbers 1–5 are used in order to indicate the stability of the athlete's psychological quality, usually using “poor performance,” “average performance,” “good performance,” “very good performance,” and “excellent performance.” The survey results are shown in Table 2.

According to the six influencing factors in the test results shown in Table 2, the chi-square test was used in turn, and the *P* value obtained in the influence of the game process exceeded 0.06, indicating that players have little influence on the results of the basketball game. In the initial, intermediate stage and final stages of the basketball game, but in the process of the basketball game, when the score is ahead, the score is behind and the score is close, the *P* value does not exceed 0.001. It shows that there is a big difference in the performance of the players in the basketball game. The *P* value corresponding to the two questions of “criticality” exceeds 0.05, indicating that the difference in the performance of the athletes is small; the *P* value corresponding to the three main questions of “psychological situation” is greater than 0.05, which also shows that these influencing factors have little effect on the athletes' competition scores.

The stability analysis function of athlete's psychological quality can be expressed by the following formula [17]:

(1) $$\begin{array}{c} O\left(x\right)=\sum_{i=1}^{\tilde{N}}\beta_{i}\left(x\right)g\left(w_{i}x_{i}+b_{i}\right). \end{array}$$

Then, it can be obtained that the corresponding weighted loss square function expression between the variable value of the output *O*_*j*_ of the function, and the expected output value of the function *t*_*j*_ is

(2) $$\begin{array}{c} E\left(x\right)=\sum_{j=1}^{N}w\left(x,x_{j}\right){\left(\sum_{i=1}^{\tilde{N}}\beta_{i}\left(x\right)g\left(w_{i}x_{i}+b_{i}\right)-t_{j}\right)}^{2}. \end{array}$$

According to the above expression, where the expression formula of the weight function is $w\left(x,x_{j}\right)=\left\{\begin{array}{cc} m^{\left(j\right)}\left(x\right), & x\in D_{j}\\ 0, & x\notin D_{j} \end{array}\right.$, then the analysis problem in the model can be converted into the solution of the minimum value in the above formula, and the expression can be obtained according to the constraints of the minimum norm:

(3) $$\begin{array}{c} \beta \left(x\right)={\left[P\left(x\right)H\right]}^{-1}P^{T}\left(x\right), \end{array}$$

where *P*(*x*)=*H*^*T*^*W*(*x*).

This study extracts the specific influencing factors *X*={*x*_1_^*n*^, *x*_2_^*n*^,…, *x*_*t*_^*n*^}, *n* ∈ [1, *N*], and N represents the specific total number of people in the scene. Assuming that *n* is 1, it represents the sequence of influencing factors in the scene. The tracked scene-level input is $\hat{X}=\left\{{\hat{x}}_{1},{\hat{x}}_{2},\ldots ,{\hat{x}}_{t}\right\}$, *P*(*x*)=*H*^*T*^*W*(*x*), and the extraction of specific static influencing factors can be calculated by the following formula :

(4) $$\begin{array}{c} I_{G}=\left(\left\{x_{1}^{1},x_{2}^{1},\ldots ,x_{T}^{1}\right\},\ldots ,\left\{x_{1}^{N},x_{2}^{N},\ldots ,x_{T}^{N}\right\},\left\{{\hat{x}}_{1},{\hat{x}}_{2},\ldots ,{\hat{x}}_{T}\right\}\right). \end{array}$$

The extraction of influence factors at the scene level can be realized by the following formula:

(5) $$\begin{array}{c} {\hat{\theta }}_{t}=f\left({\hat{X}}_{t}\right). \end{array}$$

The extraction of personal static influencing factors can be obtained through the following formula:

(6) $$\begin{array}{c} \theta_{t}^{n}=f\left(x_{t}^{n}\right). \end{array}$$

According to the test results in Figure 1, it can be seen that the scores obtained by athletes under the influence of different psychological quality stability are also sometimes high and other times low [18, 19]. Among them, the score obtained in the case of “very nervous” is the lowest, followed by “excited,” “the outside world has high expectations for the team” and “playing against teams with similar levels,” and the scores of each influencing factor can be obtained by analyzing the scores: The performance of basketball players in the three stages of “game time” is not ideal. In the stage of “mid-game,” the performance of basketball players is more prominent, and the score can reach 3.21. In the “end of the game” stage, the performance of the basketball players declined, and the score was 2.83, mainly because in the stable stage of the “middle of the game,” the basketball players played relatively stable and relaxed psychologically, so they performed relatively well. However, in the “end of the game” stage, basketball players tend to show impatience, resulting in abnormal performance of the players. According to the “game progress,” it can be concluded that in the “similar score” stage, the basketball player's performance is the worst, with a score of 2.13, and in the “outscore” stage, a value of 3.58 can be obtained through the test; The “stalemate” stage is a deadlocked condition. Both sides of the game want to widen the score gap as soon as possible, which will lead to a serious decline in the performance of the game. The scores corresponding to the “critical” questions are all very low, 2.311 and 2.229, respectively. The most important thing is that basketball players are under relatively high pressure. Under this pressure, basketball players are prone to decline, and it is especially important that the athletes are nervous. This conclusion is the same as that of many research scholars, but some basketball players have better results. According to the analysis of the “home and away” perspective, home and away games have little impact on the results of the game.

During the process of cultivating the psychological quality of basketball players, on the premise of comprehensively considering different theoretical systems and practical operations, the main training content is the training of players' attention during competition. In a basketball game, the competition between the two sides is relatively fierce. In an effective sports space, the external interference and environmental influence factors are very large. Therefore, the attention of basketball players needs to be improved. Based on cultivating athlete's attention, the athletes' different qualities such as consciousness and dynamism, alertness and persistence in the process of competition are cultivated, basketball players can grasp the adjustment methods and control of self-psychology only if they possess the above excellent quality and ability. Therefore, the cultivation of basketball players' attention can help to promote the cultivation of their psychological quality. It enables athletes to have sensitive judgment ability and field control ability in sports competitions and can make athletes make quick judgments for complex situations and changes in the course of the competition, without being disturbed by the outside world.

### 3.2. Correlation between Psychological Quality Stability and Competition Performance

After the test, the correlation degree of the relevant factors can be calculated, which can usually be expressed by the correlation coefficient. If the calculated test value is in [−1, 1], the test value greater than 0 is expressed as a positive correlation, and when it is less than 0, it is expressed as a negative correlation. The larger the absolute value of the correlation coefficient obtained by the test, the higher the degree of correlation between the influence of psychological factors. The Pearson correlation coefficient is used as a simple correlation coefficient, and the relationship between the psychological quality stability and the Pearson correlation coefficient of the game performance can be obtained as shown in Table 3.

According to the Pearson correlation coefficient value obtained from the test in Table 3, it can be concluded that the correlation between the stability of the psychological quality of different athletes and competition performance is not the same. During the “game process,” if it is in the “initial stage” and the “intermediate stage,” there is a significant positive correlation between the competition results, but there is a negative correlation between the “final stage” of the competition and the competition results. This correlation is not very strong. In the process of basketball games, the correlation between the team's “outscore” and the game performance is positive. The correlation between the game results in the “behind in the score” and “score tie” stages is negative. In the process of more important games, the results obtained in “home games” and “away games” are different, however, in the “opponent level” game, the correlation between “against a strong team” and “against a similar level” and the game performance is negative, while the correlation between “against a weak team” and the basketball game performance is positive.

Since the Pearson correlation coefficient analysis is used as a relatively simple correlation analysis method, when using the Pearson correlation coefficient for data analysis, the obtained correlation coefficient between the two variables is not only correlated with these two variables, and there are certain correlations with other variables.  Table 4 shows the partial correlation coefficient between the stability of the psychological quality of basketball players and the performance of the game.

### 3.3. Combination of Psychological Quality and Stability That Is Most Prone to Stress

The psychological tension of athletes is related to their performance in the competition. Therefore, it is necessary to pay attention to the rapid changes in the psychological quality of athletes during the competition. This is the so-called tension. How to avoid these tensions in sports competitions is the problem that researchers need exactly to solve. There are many reasons for the occurrence of tension in the game, and it is caused by many situations. What kind of combination of psychological problems is more likely to cause psychological tension? We conducted a study of some college players to analyze their psychological changes during the game. To avoid the interference of subjective factors in the player's report during the interview, such as nervousness and bad mood, the results of the judgment are affected. Therefore, our questionnaires are aimed at specific reasons. For example, the progress of the game includes the start, intermediate and end stages, as well as the score results of the games, the outscore and the lag behind in the score, as well as the analysis of the venues of the games such as home games and away games. Through the investigation and study of the stable emotional combination of basketball players under different moods, the frequency of stressful situations, the results of the questionnaire are shown in Table 5.

From the analysis results in Table 5, it can be seen from the time of the game that the closer the game is to the intermediate and the end, the more frequently the tension occurs; when the game starts, the number of times of tension is not obvious; When the score is behind and the score is the same, it is more likely to produce tension and impatience than the stage of outscores, and the occurrence of this psychological quality will interfere with the normal level of performance. Starting from the situation of home and away games, the tension in the home game is less than that in the away game. It is also based on the time of the game, especially when the score is behind and the score is tied, the home game is more prone to psychological tension., we can analyze that it is because the enthusiasm of the spectators at the home court puts a lot of pressure on the players on the scene, especially when the score is tied, when the game time enters the countdown stage, the psychological defense line of the athletes is more likely to be tensed, the pressure is doubled, and the normal level is affected. The analysis through the interference theory is that these external environments and the players' own burdens and pressures distract the concentration of the game and cause psychological tension. The questionnaire in Table 5 shows the psychologically stable combinations that generate tension. The combinations are (home game, game countdown, score tied), (home game, end time, score behind), (away game, end-stage, score behind), and (away game, end-stage, tied).

Each psychological quality and the results of the competition show different results. The factors that are more related are the three situations related to the psychological situation, all of which are related to the results of the competition, and then analyze whether it is an important competition for the two situations, including when the scores of the two sides are equal and the level is similar. Through the research on the combination of psychological quality stability, the relationship between psychological quality stability and game performance, especially in the game time period and home and away games, they have no direct correlation with the game performance. Whether the psychological quality is stable is greater than the performance coefficient of the game, which proves that the performance of the game is caused by a variety of psychological conditions. During a basketball game, it is usually because of the key operations and key stages that cause psychological pressure and psychological tension to the players. This emotion directly leads to the normal performance level of the players, resulting in abnormal performance. Especially when it comes to tit-for-tat for ball skills, high-intensity confrontation and action fouls are prone to occur, and even group fights occur. The occurrence of these situations requires psychological counseling for the athletes, improving their control, ensuring the normal progress of the game, and not affecting the psychological changes of the team due to the fierce competition and the deliberate bad actions of the opponent.

Therefore, improving the psychological quality of athletes, allowing them to maintain a rational and sober psychological quality at all times, and ensuring the normal performance of ball skills are related to the final score of the game.

## 4. Conclusion

With the continuous development of the social economy, sports have become one of the important daily necessities. Therefore, it is extremely important to focus on sports psychological quality training and improve basketball performance, especially through psychological quality training. In view of these needs and limitations, this study attempts to introduce psychological quality stability analysis. Based on the psychological quality stability model, by sorting out the psychological quality training methods of basketball players, it analyzes the effectiveness of athletes' psychological quality training in competition, and deeply analyzes the psychological factors affecting physical quality. It establishes a relationship with other psychological quality training and conducts corresponding tests to analyze the competition, realize the statistical analysis of model result calculation, aiming to analyze the effective psychological quality training program of athletes. The simulation results show that the psychological quality stability model proposed in this study is effective, has high stability and prediction accuracy, and can provide a theoretical reference for the development of men's basketball players' psychological quality, so as to further improve the performance of psychological quality training of sports.

## Figures and Tables

**Figure 1:** Comparison of athletes' performance under different psychological quality stability.

**Table 1:** Influencing factors of psychological quality stability in different basketball games.

Factor	Time variation	Competition process	Critical	Psychological fluctuation	Home game and away game	Opponent's skill
Psychological quality stability	Initial stage	Outscore	Key games	Agitation	Home game	Against strong teams
	Competition procedure	Behind in the score	Against this team	Abnormal mood	Away game	Against strong teams or weaker team
	Final stage	The score was very close	Higher expectation	Very tense		Against strong team or similar teams in level

**Table 2:** The relationship between the stability of different psychological qualities stability and the game results.

Psychological quality stability	Score
Initial stage	3.172
Intermediate stage	3.206
Final stage	2.832
Outscore	3.5824
Behind in the score	2.2618
The score was very close	2.232
Key games	2.312
The outside world has high expectations for the team	2.229
Agitation	2.026
Abnormal mood	2.264
Very tense	1.972
Home game	2.825
Away game	2.927
Against strong teams	2.657
Against weaker team	3.371
Against similar teams in level	2.243

**Table 3:** Corresponding relationship between psychological quality stability and competition performance.

Psychological quality stability	Correlation coefficient test value
Initial stage	0.255
Intermediate stage	0.388
Final stage	−0.104
Outscore	0.427
Behind in the score	−0.264
The score is similar	−0.435
Crucial game	−0.451
The outside world has high expectations for the team	−0.448
Agitation	−0.524
Abnormal mood	−0.448
Very nervous	−0.550
Home game	0.132
Away game	0.126
Against strong teams -	−0.412
Against weaker team -	0.323
Against similar teams in level	−0.525

**Table 4:** Partial correlation coefficient between psychological quality stability and competition performance.

Psychological quality stability	Correlation coefficient
Initial stage	0.032
Intermediate stage	0.045
Final stage	−0.083
Outscore	0.171
Behind in the score	−0.122
The score was very close	−0.263
Key games	−0.302
The outside world has high expectations for the team	−0.216
Agitation	−0.215
Abnormal mood	−0.237
Very nervous	−0.254
Home game	0.106
Away game	0.083
Against strong teams	−0.180
Against weaker team	0.156
Against similar teams in level	−0.216

*Notes*. ^*∗*^ means *p* < 0.05; ^*∗∗*^ means *p* < 0.01.

**Table 5:** The number of times of tension phenomenon under different combinations of psychological quality stability.

Home game		Frequency	Away game		Frequency
Initial stage	Outscore	2	Initial stage	Outscore	3
	Behind in the score	2		Behind in the score	3
	Stalemate stage	3		Stalemate stage	4
Intermediate stage	Outscore	2	Intermediate stage	Outscore	2
	Behind in the score	6		Behind in the score	4
	Stalemate stage	5		Stalemate stage	6
Final stage	Outscore	8	Final stage	Outscore	7
	Behind in the score	14		Behind in the score	12
	Stalemate stage	15		Stalemate stage	11

## Data Availability

The data used to support the findings of this study are available from the corresponding author upon request.
